The article "17β-estradiol upregulates striatin protein levels via Akt pathway in human umbilical vein endothelial cells" was retracted in 2025. Reasons: duplicated data; duplicated text; overlap with earlier publications; unreliable data.

# 17β-estradiol upregulates striatin protein levels via Akt pathway in human umbilical vein endothelial cells

**DOI:** 10.1371/journal.pone.0202500

**Published:** 2018-08-23

**Authors:** Shuhui Zheng, Peng Sun, Haimei Liu, Runmei Li, Lingli Long, Yuxia Xu, Suiqing Chen, Jinwen Xu

**Affiliations:** 1 Research Center of Translational Medicine, the First Affiliated Hospital, Sun Yat-Sen University, Guangzhou, Guangdong Province, China; 2 Department of Pathology, Sun Yat-Sen University Cancer Center, State Key Laboratory of Oncology in South China, Collaborative innovation Center for Cancer Medicine, Guangzhou, China; 3 Department of Physiology, Basic Medical College, Guangzhou University of Chinese Medicine, University Town, Guangzhou, China; 4 School of Chinese Pharmaceutical Science, Guangzhou University of Chinese Medicine, University Town, Guangzhou, China; Universita degli Studi della Campania Luigi Vanvitelli, ITALY

## Abstract

17β-estradiol (E2) has been shown to have beneficial effects on the cardiovascular system. We previously demonstrated that E2 increases striatin levels and inhibits migration in vascular smooth muscle cells. The objective of the present study was to investigate the effects of E2 on the regulation of striatin expression in human umbilical vein endothelial cells (HUVECs). We demonstrated that E2 increased striatin protein expression in a dose- and time-dependent manner in HUVECs. Pretreatment with ICI 182780 or the phosphatidylinositol-3 kinase inhibitor, wortmannin, abolished E2-mediated upregulation of striatin protein expression. Treatment with E2 resulted in Akt phosphorylation in a time-dependent manner. Moreover, silencing striatin significantly inhibited HUVEC migration, while striatin overexpression significantly promoted HUVEC migration. Finally, E2 enhanced HUVEC migration, which was inhibited by silencing striatin. In conclusion, our results demonstrated that E2-mediated upregulation of striatin promotes cell migration in HUVECs.

## Introduction

The striatin family of multidomain proteins has three members: striatin, SG2NA (striatin 3), and zinedin (striatin 4) [1–2]. These proteins contain multiple protein-binding domains: a caveolin-binding domain, a coiled-coil domain, a Ca2+-calmodulin-binding domain, and a WD-repeat domain [3]. They are involved in Ca2+-dependent pathways by binding calmodulin in the presence of Ca2+ ions, and interact with caveolin [4]. Striatin, a cytoplasmic protein, was identified in brain tissue, and is detectable in liver, skeletal muscle, the heart, and vascular cells [4–9]. A previous study demonstrated that a polymorphic variant in the striatin gene is associated with salt-sensitive blood pressure (BP) in people with hypertension. Striatin heterozygous knockout mice also demonstrate salt sensitivity of BP [10]. Furthermore, striatin deficiency was found to increase vasoconstriction and decrease vascular relaxation [11]. These results suggest that striatin might regulate vascular function.

Estrogen has been shown to regulate cardiovascular function though genomic and nongenomic mechanisms [12–13]. The genomic effects of estrogen are mediated by nuclear estrogen receptors (ERs) that act as ligand-activated transcription factors. The nongenomic effects of estrogen are also mediated by ERs, although they occur relatively quickly and do not involve alterations in gene expression. In vascular endothelial cells, the nongenomic effects of estrogen were found to be associated with striatin [14]. Moreover, we previously showed that estrogen upregulates the expression of striatin, and inhibits cell migration in vascular smooth muscle cells [9]. The objective of the present study was to investigate the effects of estrogen on striatin expression in human umbilical vein endothelial cells (HUVECs).

## Methods

### Reagents

17β-Estradiol (E2), PD98059, and wortmannin were from Sigma-Aldrich (St. Louis, MO). ICI 182780 was from Tocris Cookson (Bristol, UK). Dulbecco’s modified Eagle’s medium (DMEM), Opti-MEM, and fetal bovine serum (FBS) were from Invitrogen (Carlsbad, CA). All other chemicals were of analytical grade and from Guangzhou Chemical Reagents (Guangzhou, China).

### Cell culture

Human umbilical vein endothelial cells were cultured as previously described [15]. Cells were grown in a 5% CO2 atmosphere at 37°C in DMEM without phenol, supplemented with penicillin and streptomycin, and 10% charcoal-stripped FBS (steroid free and delipidated, fetal bovine serum) (Biowest, S181F-500, Nuaille, France). Before experiments, cells were maintained in phenol red-free DMEM containing 1% FBS for 48 h. Chemical inhibitors were added to cells 30 min before starting other treatments.

### Immunoblotting

Immunoblotting was performed as previously described [9]. Briefly, HUVECs in culture dishes maintained on ice were rinsed once with ice-cold phosphate-buffered saline before the addition of lysis buffer (100 mM Tris-HCl, pH 6.8, 4% sodium dodecyl sulfate, 20% glycerol, 1 mM sodium orthovanadate, 1 mM NaF, and 1 mM phenylmethylsulfonyl fluoride). Cell lysates were separated by sodium dodecyl sulfate-polyacrylamide gel electrophoresis. The antibodies used were: striatin (BD Transduction Laboratories), Akt, and Ser 473 phosphorylated Akt (Cell Signaling Technology). Membranes were incubated with primary and secondary antibodies using standard techniques. Immunodetection was performed using enhanced chemiluminescence.

### Immunofluorescence

HUVECs were grown on coverslips and treated accordingly. Cells were fixed with 4% paraformaldehyde and permeabilized with 0.1% Triton-X. Blocking was performed with 3% normal serum for 20 min. Cells were incubated with an antibody against striatin (BD Transduction Laboratories) and a FITC-conjugated secondary antibody (K00018968, Dako North America Inc., Dako, Denmark). After washing, the nuclei were counterstained with 4′-6-diamidino-2-phenylindole (Sigma). Immunofluorescence was visualized using an Olympus BX41 microscope (Tokyo, Japan) and recorded with a high-resolution DP70 Olympus digital camera.

### Transfection experiments

Transfection experiments were performed as previously described [9]. Striatin siRNAs, including siRNA1 (SASI_Rn01_00107865), siRNA2 (SASI_Rn02_00266690), and siRNA3 (SASI_Rn01_00107867) were purchased from Origene. They were transfected into HUVECs using lipofectamine according to the manufacturer’s protocol. Cells (40% confluent) were serum-starved for 1 h, followed by incubation with 100 nM target siRNA or control siRNA for 6 h in serum-free media. Media supplemented with serum (10% final concentration) was then added for 42 h before experiments and/or functional assays were performed. Target protein silencing was assessed through immunoblotting up to 48 h after transfection.

For striatin overexpression assays, each plasmid (15 mg) was transfected into HUVECs using the Lipofectamine (Invitrogen) according to the manufacturer’s instructions. The transfected plasmids were as follows: overexpressed striatin plasmid and empty pcDNA3.1+ plasmid. These constructs were obtained from Genechem Co.Ltd. (Shanghai, China). All the inserts were cloned in pcDNA3.1+. As control, parallel cells were transfected with empty pcDNA3.1+ plasmid encoding a enhanced green fluorescent protein(EGFP). And the transfection efficiency was quantified by counting the percentage of cells that EGFP-positive using a microscope. Cells (60–70% confluent) were treated 24 h after transfection, and cellular extracts were prepared according to the experiments to be performed.

### Cell migration and transwell assays

Cell migration was assayed as previously described [16–17]. Briefly, after transfection with siRNA, HUVECs were synchronized by replacing media with serum-free DMEM for 24 h. To create wounds, cell monolayers in culture dishes were scratched with 200-μl pipet tips. Cells were washed, and DMEM medium containing gelatin (1mg/mL) and cytosine b-D-arabinofuranoside hydrochloride (Ara-C, Sigma) (10mM), a selective inhibitor of DNA synthesis which does not inhibit RNA synthesis, was added. Migration was monitored for 24 h. Cells were imaged digitally with phase-contrast microscopy, and migration was quantified as the extent of gap closure using NIH Image J software (Bethesda, MD).

Transwell experiments were performed as previously described [18]. After transfection with the different siRNAs, cells were seeded in the upper chamber of transwell chambers (Corning Life Sciences, Lowell, MA, USA) and Ara-C (10 μM) was added. After 24 h, cells that invaded the lower surface of the membranes were fixed with methanol for 10 min, and stained with hematoxylin. The cells on the lower side of the membrane were counted and averaged in six high-power fields with a light microscope.

### Statistical analysis

Data are presented as mean ± standard deviation, and represent at least three independent experiments. Statistical comparisons were made using the Student’s t-test or one-way analysis of variance followed by a post hoc analysis (Tukey test) where applicable to identify significant differences in mean values. p<0.05 was considered statistically significant.

## Results

### E2 increases striatin protein expression in HUVECs

Immunoblotting showed that E2 (0.1nM–1.0μM) upregulated striatin expression with the maximal effect achieved using 10 nM E2 (Fig 1A). Furthermore, E2 (10 nM) increased striatin expression in a time-dependent manner within 48 h (Fig 1B). Immunofluorescence consistently demonstrated that treatment with 10 nM E2 for 24 h increased cytoplasmic striatin protein expression in HUVECs (Fig 1C).

**Fig 1:** E2 upregulated striatin expression in HUVECs. (A) and (B) show the dose- and time-dependent striatin protein expression in HUVECs after treatment with E2. Striatin densitometry values were adjusted to actin intensity, then normalized to expression from the control sample. Expression in CON group was normalized to 1, *p<0.01 versus CON. Bars represent SD, n = 4. (C) HUVECs were treated with E2 (10nM) for 24h. Then the cells were stained with anti-striatin linked to FITC. Nuclei were counterstained with DAPI.

### E2 increases striatin protein expression via the Akt pathway

To determine the signaling pathways involved in E2-induced upregulation of striatin expression, HUVECs were pretreated with the mitogen-activated protein kinase inhibitor, PD98059, the phosphatidylinositol-3 kinase inhibitor, wortmannin, and the Src inhibitor, PP2. We found that wortmannin inhibited E2-induced striatin protein expression (Fig 2A). We furthermore found this inhibitory effect of wortmannin was in a dose manner (Fig 2B). Treatment with E2 resulted in Akt phosphorylation (Ser 473) from 5 min to 30min (Fig 2C).

**Fig 2:** E2 upregulated striatin expression via Akt pathway in HUVECs. **(**A) HUVECs were treated with E2 (10nM) for 24h, in the presence or absence of the pure ER antagonist ICI 182,780 (ICI– 1mM), of the MEK inhibitor PD98059 (PD– 5mM), of the PI3K inhibitor wortmannin (WM– 30nM) or of the c-Src kinase inhibitor, PP2 (10mM). Striatin densitometry values were adjusted to actin intensity, then normalized to expression from the control sample. Expression in CON group was normalized to 1, *p<0.01 versus CON, **p<0.01 versus E2. Bars represent SD, n = 4. (B) HUVECs were treated with E2 (10nM) for 24h, in the presence of the PI3K inhibitor wortmannin (WM –5- 30nM). Striatin densitometry values were adjusted to actin intensity, then normalized to expression from the control sample. Expression in CON group was normalized to 1, *p<0.01 versus CON, **p<0.01 versus E2. Bars represent SD, n = 4. (C) HUVECs were treated with E2 (10nM) for the indicated time and wild-type Akt or Ser 473-phosphorylated Akt (p-Akt) were detected by western blot. p-Akt densitometry values were adjusted to Akt intensity, then normalized to expression from the control sample. Expression in CON group was normalized to 1, *p<0.01 versus CON. Bars represent SD, n = 4.

### Silencing striatin in HUVECs inhibites cell migration

When transfected with striatin siRNAs, striatin expression was significantly reduced (Fig 3A). Silencing striatin increased HUVEC gap distance by approximately 180% (Fig 3B). Consistently, transwell experiments showed that silencing striatin significantly reduced the number of cells that invaded the lower surface of the membranes by 60% (Fig 3C).

**Fig 3:** Silencing striatin in HUVECs inhibites cell migration. (A) HUVECs were transfected with scrambled siRNA or striatin targeted siRNA 1, 2 or 3 for 48h. Striatin densitometry values were adjusted to actin intensity, then normalized to expression from the control sample. Expression in CON group was normalized to 1, *p<0.01 versus CON. Bars represent SD, n = 4. (B) After transfection assays, HUVECs were scrapped to create a cell-free (wounded) area. Cells were incubated with 10nM E2 or with solvent as control for another 24h. Migration was monitored. Representative images of cell migration are shown. Gap distance in CON group was normalized to 1, *p<0.01 versus CON. Bars represent SD, n = 6. (C) After transfected with striatin siRNA1, 2, 3 or scrambled siRNA for 24h, transwell experiments were performed. Representative images of transwell experiments are shown. The number of the invaded cell in the lower surface of the membrane in CON group was normalized to 1, *p<0.01 versus CON. Bars represent SD, n = 6.

### Striatin overexpression in HUVECs promotes cell migration

When transfected with plasmid striatin, striatin expression was significantly increased (Fig 4A). Striatin overexpression decreased HUVEC gap distance (Fig 4B). Consistently, transwell experiments showed that striatin overexpression significantly increased the number of cells that invaded the lower surface of the membranes by approximately 100% (Fig 4C).

**Fig 4:** Striatin overexpression in HUVECs promotes cell migration. (A) HUVECs were transfected with control plasmids (PL-con) or striatin targeted plasmids (PL-striatin). Striatin densitometry values were adjusted to actin intensity, then normalized to expression from the control sample. Expression in PL-con group was normalized to 1, *p<0.01 versus CON. Bars represent SD, n = 4. (B) After transfection assays, HUVECs were scrapped to create a cell-free (wounded) area. Migration was monitored. Representative images of cell migration are shown. Gap distance in PL-con group was normalized to 1, *p<0.01 versus CON. Bars represent SD, n = 6. (C) After transfected with striatin plasmids, transwell experiments were performed. Representative images of transwell experiments are shown. The number of the invaded cell in the lower surface of the membrane in PL-con group was normalized to 1, *p<0.01 versus CON. Bars represent SD, n = 6.

### E2 promotes HUVEC migration via striatin

Next, we explored the effects of striatin on E2-induced cell migration in HUVECs. E2 significantly decreased HUVEC gap distance by 50% (Fig 5), and increased the number of cells that migrated to the membrane by 90% (Fig 6). These results indicated that E2 increases HUVECs migration. However, after transfected with siRNAs, E2-induced cell migration distance and the number of migrated cells were significantly reduced (Figs 5 and 6).

**Fig 5:** Wound scratch assay showed E2 promotes HUVEC migration via striatin. HUVECs were transfected with striatin siRNA1, 2, 3 or scrambled siRNA for 24h. Then cells were scrapped to create a cell-free (wounded) area. Cells were incubated with 10nM E2 or with solvent as control for another 24h. Migration was monitored. Representative images of cell migration are shown. Gap distance in CON group was normalized to 1, *p<0.01 versus CON. Bars represent SD, n = 6.

**Fig 6:** Transwell assay showed E2 promotes HUVEC migration via striatin. After transfected with striatin siRNA1, 2, 3 or scrambled siRNA for 24h, transwell experiments were performed. Representative images of transwell experiments are shown. The number of the invaded cell in the lower surface of the membrane in CON group was normalized to 1, *p<0.01 versus CON. Bars represent SD, n = 6.

## Discussion

The striatin scaffold proteins interact with signaling proteins, including members of the germinal center kinase family (MST3, MST4, and YSK1), NCK-interacting kinase (NIK), and TRAF2- and NCK-interacting kinase (TNIK) [19]. The protein complex, striatin interacting phosphatase and kinase (STRIPAK), acts as a signaling hub that regulates multiple cellular functions [2]. Although the nongenomic effects of E2 on vascular endothelial cells have been shown to be regulated by striatin [14], little is known about the effects of E2 on striatin expression in endothelial cells. Furthermore, a previous study showed that incubation of EA.hy926 endothelial cells with aldosterone increases striatin protein and mRNA expression [20]. We previously demonstrated that E2 increases striatin protein levels in vascular smooth muscle cells (VSMCs) [9]. Therefore, we hypothesized that E2 regulates striatin expression in HUVECs. We found that E2 (0.1nM–1.0μM) significantly upregulated striatin expression in HUVECs (Fig 1). Immunofluorescence further confirmed that cytoplasmic striatin expression was increased in response to treatment with E2 (Fig 1).

To determine the signaling pathways involved in E2-induced upregulation of striatin, we treated HUVECs with several signal transduction inhibitors. We previously showed that ERK1/2 is involved in E2-induced upregulation of striatin in VSMCs [9]. However, in the present study, we found that wortmannin suppressed E2-induced upregulation of striatin expression in HUVECs, while PP2 and PD98059 had no effects (Fig 2). Previously found that estrogen induced rapid activation of Akt in EA.hy926 endothelial cells [21]. Herein, we consistently found that treatment with 10 nM E2 resulted in Akt phosphorylation within 5 min (Fig 2). These results indicated that E2 upregulates striatin via the Akt pathway in HUVECs. Interestingly, striatin was found to play a role in the estrogen-induced rapid activation of Akt in EA.hy926 endothelial cells [14]. These observations suggest striatin may be involved in crosstalk between the genomic and nongenomic effects of E2 in HUVECs.

Cardiovascular disease is less frequent in premenopausal women compared with men, but increases rapidly in postmenopausal women [22]. Although the primary results from the Women’s Health Initiative showed no cardiovascular benefit from estrogen replacement therapy [23], the Danish Osteoporosis Prevention Study showed that women who received hormone replacement therapy early after menopause had a significantly reduced risk of mortality, heart failure, or myocardial infarction [24]. This beneficial effect of E2 on the cardiovascular system was shown to be associated with accelerated vascular endothelial repair through the promotion of endothelial migration [25–26]. In cell culture, E2 has been shown to promote the growth and migration of vascular endothelial cells, an essential component of vascular healing [27–28]. It was found that silencing striatin 4 suppresses cell migration in several cancer cell lines [29]. We assumed that E2-induced up-regulation of striatin might affect cell migration in HUVECs. We furthermore found that striatin overexpression significantly increased cell migration in HUVECs, while, striatin silencing reduced cell migration. However, previous study demonstrated that E2 in vitro directly promoted HUVECs migration [30]. Our results indicated E2-induced cell migration in HUVECs might partially through up-regulation of striatin expression. Finally, with cell migration and transwell assays, we demonstrated that silencing striatin in HUVECs significantly inhibited E2-induced cell migration.

## Conclusions

In conclusion, our findings indicated that E2-induced cell migration may be associated with upregulation of striatin in HUVECs.

## Supporting information

S1 Data All relevant raw data are within RAW DATA.pptx files. (PPTX)
